The article "Bioflavonoid Galangin Suppresses Hypertrophic Scar Formation by the TGF-β/Smad Signaling Pathway" was published in 2021. Journal: Evid Based Complement Alternat Med.

# Bioflavonoid *Galangin* Suppresses Hypertrophic Scar Formation by the TGF-*β*/Smad Signaling Pathway

**DOI:** 10.1155/2021/2444839

**Published:** 2021-09-04

**Authors:** Zha Ru, Ying Hu, Shenghua Huang, Li Bai, Kun Zhang, Yue Li

**Affiliations:** ^1^Department of Plastic Surgery, The Third Affiliated Hospital of Sun Yat-Sen University, Guangzhou 510630, China; ^2^Department of Traditional Chinese Medicine, The Third Affiliated Hospital of Sun Yat-Sen University, Guangzhou 510630, China

## Abstract

**Background:**

Hypertrophic scar (HS) is a benign fibroproliferative skin disease resulting from an aberrant wound healing process and can cause aesthetic and functional damage to patients. Currently, there is no ideal treatment to treat this disease. *Galangin*, a natural active bioflavonoid compound, is suggested to inhibit fibrosis and proliferation in certain cells.

**Methods:**

In this study, we found *Galangin* could attenuate abnormal scar formation in an HS rabbit ear model. Additionally, the HE staining shows *Galangin* reduced scar elevation index (SEI) and Masson's trichrome staining changed collagen deposition.

**Results:**

The expressions of type I collagen, type III collagen, and TGF-*β*1 were much lower under a proper dose of *Galangin* treatment, and Smad7 expression was also enhanced, which are examined by real-time PCR, immunohistochemistry, and western blot.

**Conclusion:**

Our data indicated that *Galangin* can alleviate dermal scarring via the TGF-*β*/Smad signaling pathway probably by upregulating Smad 7 expression and, thus, suppressing the expression of type I and type III collagens and TGF-*β*1.

## 1. Background

Scarring is an inevitable natural process during wound healing. The wound healing progress is a complex one which involves many types of cells, mediators, and three sequential steps: inflammation, new tissue formation, and remodeling [1, 2]. Besides, the remodeling phase comes with scar formation to some extent. However, in some cases, hypertrophic scar (HS) is formed, which is defined as an excessive scar tissue within the original wound. Despite the yet unknown detailed mechanism of HS, some factors are considered to be related to HS formation, such as age, bacterial colonization, and skin stretch [3, 4]. Collagen is overdeposited in the extracellular matrix (ECM), and the fibroblasts become overproliferated during the remodeling phase of wound healing [5]. As a result, wound healing ends up with HS formation, which may cause dysfunction, pain, aesthetic problem, etc. [6]. Although several decades have been spent to searching optimal treatments for HS, it remains an unmet challenge.

However, unlike the scar formation in adults, wound healing of fetal tissue is scarless [7]. The expression of cytokines, growth factors, and ECM deposition in the injured tissue differs significantly, among which transforming growth factor-*β* (TGF-*β*) is considered to play the key role [8]. TGF-*β*, activated by Smad proteins in fibroblasts, interacts with TGF-*β* receptor and leads to an increase in the production of collagen in the ECM and cell proliferation [9]. Smad 7, as the particularly negative feedback regulator of the TGF-*β*/Smad signal path, can prevent receptor-regulated Smads (*R*-Smads) phosphorylation by integrating with the activated TGF-*β*1 receptors. Therefore, an overexpression of Smad 7 may possibly attenuate TGF-*β*1 excretion and inhibit fibrinolysis [10].

*Galangin* is a flavonoid compound extracted from Chinese galangal root and used as herbal treatment in traditional medicine, which is also used in modern clinical treatment because of its antioxidant, anti-inflammatory, and proapoptosis effects [11–13]. Also, the bioflavonoid had been reported of its alleviating fibrosis effect in the kidney and renal organs [14, 15]. Considering the bioactivity and pharmacological effects of *Galangin*, we wondered whether it can be used to inhibit HS formation in vivo. Besides, among a large amount of studies to investigate the therapeutic effect of bioflavonoid, little is known about its effect in HS formation.

In this study, HS models were established in rabbits' ears. The effect of bioflavonoid on HS was investigated, and its unique role in regulating the expression of key factors in the TGF-*β*/Smad signaling pathway was studied.

## 2. Materials and Methods

### 2.1. Animals

All procedures of this experiment were approved by the Ethics Committee of the First Affiliated Hospital of Xinjiang Medical University. Also, our researchers observed the Animal Welfare Act. Twenty female New Zealand white rabbits (weighing 2.0 to 2.8 kg, cleaning I grade) were single-housed under the same standard in the Laboratory Animal Center of Xinjiang Medical University (License No. 20170214-71).

### 2.2. Preparation of Rabbit Ear HS Models, Treatment, and Sampling

On day 0, rabbits were anesthetized by intramuscular injection with 0.15 mL/kg Zoletil 50 (tiletamine hydrochloride and zolazepam hydrochloride) and 0.1 mL/kg ketamine, respectively. Under sterile conditions, six 8 mm diameter round full-thickness dermal wounds were excised down to the bare cartilage on the ventral surface of each ear [16]. The bare cartilages, from the epidermis to perichondrium, were all removed under a surgical operating microscope [17]. During the excision, visible vessels were avoided and bleeding was treated by manually pressing with gauze. All of the wounds were then banded with sterile adhesive dressings. A total of 240 wounds were created in 20 rabbits. On day 15, successfully established HS models were divided into four groups along the vertical axis of each ear from left to right in 19 rabbits (one rabbit died on day 2 probably due to the anesthetization side effects) (Figure 1). Subsequently, 219 HSs (9 scars were excluded because of invagination) were treated by intralesional injection of either normal saline (group *A*, *n* = 55) or different doses of *Galangin* solution (group *B*, *n* = 54, 2 mg/mL; group *C*, *n* = 56, 1 mg/mL; and group *D*, *n* = 54, 0.5 mg/mL), which were purchased from Shanxi Guanchen Biotechnology Co., Ltd., China (GC-01-398, Purity:  ≥ 98% (HPLC)) and ultrasonic dissolved with normal saline [16, 18]. The injection was performed every three days and four times in total. In addition, since day 15 after wounding, photographs of ears and scarring areas were taken before each time of injection for qualitative changes in scar morphology [19]. On day 27, rabbits were sacrificed and 207 HS tissue (a rabbit died after the second injection) were harvested with a 3 mm unwounded margin (Figure 1(e)). From each group, 45 HSs were randomly collected.

### 2.3. Histopathological Analysis

The 60 HSs (15 in each group) were fixed with formaldehyde, embedded in paraffin, cut into 4 *μ*m sections, and stained for histopathological analysis. After haematoxylin and eosin (HE) stain, the protuberant degrees were measured as scar elevation index (SEI), which represents the ratio of the scar area to the estimated area below the protuberant portion that had the neogenesis with the same height as the surrounding nonwounded dermis [16]. To analyze collagen deposition and arrangement, Masson's trichrome staining was carried out using a quick staining kit (Njjcbio, China) as the manufacturer's instruction recommended. For immunohistochemistry, the endogenous peroxidase was inactivated by 3% H_2_O_2_ incubation for 10 minutes at around 25°C, and then, the sections were incubated with 1% citric acid for 10 minutes in a microwave for antigen retrieval. After that, the sections were blocked with normal goat serum (ZSGB-Bio, China) for 15 minutes at 37°C and then incubated with primary antibodies of collagen I (Cat# ab90395; 1 : 1000dilution; Abcam), collagen III (Cat# ab7778; 1 : 5000 dilution; Abcam), TGF-*β*1 (Cat# sc-146; 1 : 500 dilution; Santa Cruz Biotechnology), and Smad-7 (Cat#sc-365846; 1 : 500 dilution; Santa Cruz Biotechnology) at 4°C overnight. Finally, sections were incubated with goat anti-rabbit secondary antibody (Boster, China) or goat anti-mouse secondary antibody (Boster, China) for 30 minutes at 37°C, followed by DAB (Boster, China) coloration for 5 minutes and haematoxylin staining. All histological images were obtained with an optical microscope connected to cellSens software (Olympus, Japan), and the quantification of positive cells in immunohistochemistry was carried out using Image J software (1.52 v).

### 2.4. Real-Time PCR

Sixty (15 for each group) HS samples were ground into powders in liquid nitrogen, and then, total RNA was extracted using TRIzol® (Invitrogen) following the manufacturer's instructions. RNA was reverse-transcripted into cDNA with a RevetAid First Strand cDNA Synthesis Kit (Thermo Scientific, USA). Real-time PCR was operated using the Maxima SYBR Green qPCR Master Mix (Thermo Scientific, USA) on the iQCycler thermocycler (Bio-Rad). The primer sequences (synthesized by Sangon Biotech, China) are listed in Table 1. Real-time PCR was carried out as follows: initial denaturation for 10 minutes at 95°C and 40 cycles of 15 seconds at 95°C and 60 seconds at 60°C. Quantification was always normalized to the internal control GAPDH, and each template was repeated three times under the same condition.

### 2.5. Western Blot

Briefly, 60 HS tissue samples (15 each group) were lysed with Pierce® RIPA buffer (Thermo Scientific, USA) and PMSF (100 : 1). The extracted proteins were measured by using the Pierce® BCA Protein Assay Kit (Thermo Scientific, USA). Proteins were isolated on 12% SDS-PAGE and transferred to polyvinylidene fluoride (PVDF) membranes (Millipore, Bedford, USA). Then, the membranes were incubated with primary antibodies of collagen I (Cat# ab90395; 1 : 500 dilution; Abcam), collagen III (Cat# ab7778; 1 : 1000 dilution; Abcam), TGF-*β*1 (Cat# sc-146; 1 : 200 dilution; Abcam), Smad-7 (Cat# sc-365846; 1 : 200 dilution; Abcam), and *β*-actin (Cat# sc-47778; 1 : 500 dilution; Santa Cruz Biotechnology) overnight at 4°C, respectively. After PBS washing, HRP-conjugated goat anti-rabbit or goat anti-mouse secondary antibody (Abbkine, USA) was added and incubated at around 25°C for 2 hours. The protein bands were visualized using the ECL Kit (Thermo Scientific, USA), and the densities of the bands were compared with that of *β*-actin as reference.

### 2.6. Statistical Analysis

All statistic data were analyzed with SPSS version 22 and were demonstreated as mean ± standard deviation (SD). Intergroup comparisons were analyzed by Student's *t*-test. One-way ANOVA was used to compare the mean values of four groups simultaneously, followed by Tukey's test or Tamhane's method while the variance was not homogenous. *P* value less than 0.05 was considered as statistically significant.

## 3. Results

### 3.1. Effect of *Galangin* on Gross Scar Formation

To dynamically observe the scar-forming progress and the effect of *Galangin* on scar formation since day 15 after wounding (Figure 1(a)), the scars were observed every day and photographed before each injection. The intralesional *Galangin* injection groups showed obvious softness after the second injection compared with the control group (Figure 1(b)). Some HSs in group *C* and *D* almost resembled the normal skin, which had lower protuberant heights (Figure 1(c)). Some vulnerable epidermis samples were observed in group *B*, in the form of bleeding or ulceration. In addition, a rabbit showed slouched ears because of the scar contracture, but the sides of rabbit ears in group *C* and *D* became erected again after the third injection (Figure 1(d)). These results indicate that *Galangin* may soften the scar and delay the wound healing.

### 3.2. Effect of *Galangin* on SEI and Collagen

To evaluate the effects of *Galangin* on cell morphology, HE staining was performed. Many spindle-shaped cells of the control group were observed, while most of them in the *Galangin* injection groups were round. The number of fibroblasts was the lowest in group *C* (Figure 2(a)). Furthermore, the quantitative analysis of SEI decreased from 1.75 ± 0.13 to 1.68 ± 0.08, 1.57 ± 0.10, and 1.58 ± 0.86 (Figure 2(b)). These results suggest that treatment with a proper dose of *Galangin* may restrain the proliferation of fibroblasts and less decrease the protuberant degree of HSs. The HS tissues were subjected to Masson staining to examine the effect of *Galangin* on collagen arrangement. It showed that the collagen was sparsely distributed and arranged as a net-like shape resembling to the surrounding unwounded tissues in the *Galangin*-treated groups, especially in group *C* and *D*, while the collagen of the control group was densely arranged, parallel to the epithelium and less mature with more fibroblasts (Figure 2(c)). Therefore, treatment with a proper dose of *Galangin* may lead to collagen arranging and depositing in a beneficial direction.

### 3.3. The Effect of *Galangin* on the Protein Expressions of Type I Collagens, Type III Collagens, TGF-*β*1, and Smad 7

In order to observe the expression of type I collagens, type III collagens, TGF-*β*1, and Smad 7 of HS tissues, immunohistochemical staining was performed. There was less type I collagen deposition in the cellular mesenchyme after *Galangin* treatment from 10.97 ± 0.53 to 6.24 ± 0.60, 4.12 ± 0.65, and 4.21 ± 0.54 (Figure 3(a), *E*, *P* < 0.05), and type III collagen deposition also decreased from 16.84 ± 0.42 to 13.71 ± 0.47, 11.79 ± 0.60, and 8.83 ± 0.56 (Figure 3(b), *F*, *P* < 0.05). Besides, expressions of TGF-*β*1 were 15.14 ± 0.71, 17.10 ± 0.36, 12.34 ± 0.73, and 10.88 ± 0.63 (Figure 3(c), *G*, *P* < 0.05), and a higher expression was detected in group B. Also, Smad 7 increased in the *Galangin*-treated groups, from 4.33 ± 0.26 to 5.47 ± 0.41, 6.81 ± 0.46, and 11.45 ± 0.56 (Figure 3(d), *H*, *P* < 0.05). To further verify the influence of *Galangin* treatment on the protein expressions of type I collagens, type III collagens, TGF-*β*1, and Smad 7, western blot was performed. The results demonstrated that type I collagens and type III collagen expressions remarkably reduced in the *Galangin*-treated groups from 1.32 ± 0.09 to 0.83 ± 0.21, 0.27 ± 0.12, and 0.34 ± 0.16 and from 1.27 ± 0.02 to 0.90 ± 0.09, 0.65 ± 0.11, and 0.34 ± 0.09, respectively (Figures 4(b) and 4(c), *P* < 0.05). The TGF-*β*1 protein expressions were 1.13 ± 0.27, 1.56 ± 0.09, 0.36 ± 0.07, and 0.16 ± 0.05, which were effectively suppressed in group *C* and *D*, while a higher expression was detected in group *B* (Figure 4(d)*P* < 0.05). By contrast, the Smad 7 protein expression significantly increased after *Galangin* treatment, from 0.18 ± 0.08 to 0.46 ± 0.25, 0.81 ± 0.13, and 1.21 ± 0.11 (Figure 4(d), *P* < 0.05). Thus, it is assumed that *Galangin* might reduce collagen deposition and TGF-*β*1 expression, while promoting Smad 7 expression.

### 3.4. The Effect of *Galangin* on the mRNA Expressions of Type I Collagens and Type III Collagens, TGF-*β*1, and Smad 7

To test the mRNA expressions of type I collagens and type III collagens, TGF-*β*1, and Smad 7, quantitative RT-PCR was carried out. The results demonstrated that the type I collagen mRNA expression was suppressed in all the *Galangin*-treated groups (Figure 5(a), *P* < 0.05), especially in group *C* (*Galangin*, 1 mg/mL). The mRNA expressing of type III collagen and TGF-*β*1 was inhibited in the *Galangin*-treated groups, among which the effect in group *D* (*Galangin*, 0.5 mg/mL) was the most significant (Figures 5(b) and 5(c), *P* < 0.05). In contrast, the mRNA expression of Smad 7, which is considered as a unique inhibitor of the TGF-*β*/Smad signal pathway, in the *Galangin*-treated groups was much higher than that of the control group (Figure 5(d), *P* < 0.05). These results suggest that the mRNA levels of type I collagen and type III collagen and TGF-*β*1 were downregulated after a proper dose of *Galangin* treatment, while the Smad 7 level was upregulated.

## 4. Discussion

Scar formation is the normal consequence of skin injury, which is thin and resembles normal skin under correct regulation. However, prolonged inflammation, local mechanical tension, and chronic stimulation may cause excessive deposition of collagen and proliferation of fibroblasts, eventually leading to HS formation [9, 10, 20]. Moreover, because of the overproliferated and overactivated fibroblasts, HS also is considered as a benign skin tumor [21]. So far, although the treatment for HS is still unsatisfying, surgical operation to reduce local force and anti-inflammatory and anti-angiogenesis treatment are applicable strategies [22]. *Galangin*, a kind of bioflavonoid, is found to have antiproliferative property to certain cells [11, 23, 24]. Besides, bioflavonoid has also been proved to alleviate fibrosis in the liver [15]. Thus, based on the abovementioned study, we assumed that *Galangin* could suppress HS formation, and this assumption is proved in our further investigation which shows that *Galangin* could soften the HSs and decrease the SEI of the rabbit ear model in vivo.

Previous studies have suggested that wound healing and scarring are closely related to TGF-*β* family members, which also participate in regulations of a wide spectrum of cellular functions such as proliferation, differentiation, migration, and apoptosis [25, 26]. Increased amounts of TGF-*β* have been found in HS, and the scar-free healing in human fetus is considered as a consequence of TGF-*β* deficiency [8, 27]. Besides, it has been reported that TGF-*β* mediates the fibroblast proliferation, angiogenesis, ECM synthesis, and reepithelialization during the wound healing course [28, 29]. Overexpression of TGF-*β*1 and TGF-*β*2 was detected in HSs, whereas TGF-*β*3 was reported to have antifibrotic effects [10]. Particularly, TGF-*β*1 regulates various fibrosis-related proteins transcriptionally, including type I collagen and type III collagen [30, 31]. A previous study showed that bioflavonoid can attenuate TGF-*β*-induced fibrosis in human tubular epithelial cells [14]. Also, our preliminary study in vitro shows that bioflavonoid dose-dependently decreased cell viability in fibroblast cells [32], and the high expression of TGF-*β*1 protein in group *B* (*Galangin*, 2 mg/mL) might be due to the high dose of bioflavonoid which may cause tissue damage, though no visible wounds were observed on rabbit ears; thus, the proper dose of *Galangin* in vivo and toxicity study for epidermal cells need further tests. It can also accelerate the transformation of fibroblasts to myofibroblasts, which are considered as major cells in HS formation and characterized as an improved propensity to synthesize collagen and upregulation of cytokines [33, 34]. Therefore, it is speculated that attenuation of TGF-*β*1 activities would have potential advantages in inhibiting HS formation.

Despite the limited varieties of TGF-*β* receptors and Smads, there may be a greater variety of the signal possibilities than we used to expect. Combinatorial interactions between TGF-*β* receptors and Smads in oligomeric complexes allow substantial diversity and are complemented by various sequence transcription factors cooperating with Smads, leading to context-dependent transcriptional regulation [35–37]. Additionally, other signaling pathways may also help to define the responses to TGF-*β*, and it is evidently shown that TGF-*β*-related protein activation is not a linear signaling transduction pathway. These pathways not only involve Smad-dependent responses but also the Smad-independent responses [38]. On the one hand, the TGF-*β*1-activated Smad-dependent pathways can cause cellular changes such as the collagen synthesis and secretion, leading to the aggravated scar formation. However, Smad-independent signaling paths may improve healing. Therefore, inhibition of TGF-*β*1 transcription may reduce scarring but delay wound healing [39–41]. In the current study, it was observed that treatment with a proper dose of *Galangin* could lessen scarring and delay healing. Meanwhile, the Smad 7 expression was upregulated and that of TGF-*β*1 was decreased.

There are three distinct Smad subfamilies: receptor-regulated Smads (*R*-Smads), common-partner Smads (Co-Smads), and inhibitory Smads (I-Smads). Smad 7, which acts as the I-Smads of TGF-*β* family signaling, can bind with TGF-*β* receptor, thus preventing the recruitment and phosphorylation of effector Smads and inhibiting TGF-*β*/Smads signaling [10, 38, 42]. The TGF-*β*/Smad signal path is an autoinhibitory loop to control the intensity and duration of TGF-*β* signaling response. TGF-*β* stimulation could cause the export of Smad 7 from the nucleus [37]. Therefore, the expression level of Smad 7 will influence TGF-*β* transcriptional responses. Cells with a higher level of Smad 7 are more inclined to resist the profibrotic activities of TGF-*β*. As this study indicated, *Galangin* treatment blocked the TGF-*β*/Smad signaling via increasing the expression of Smad 7, and thus, the stimulation effect of TGF-*β*1 on collagen deposition in ECM was inhibited.

## 5. Conclusions

The rabbit ear HS model was established successfully. A proper dose of *Galangin* could negatively regulate the expression of type I collagens and type III collagens and the collagen deposition. TGF-*β*1 transcription was downregulated, which might be partially due to Smad 7 upregulation. This study suggests that *Galangin* may have potential to prevent HS formation.

## Figures and Tables

**Figure 1:** Gross images of representative scarring samples. (a) On day 15 after wounding, the epithelialization was completed and the HS model was accomplished. (b) After the second injection (day 20), the HSs in group *C* and *D* were more softened and had lower protuberant heights. (c) At the end of the injection (day 27), a much more significant effect in the *Galangin* injection groups was observed. G. A : group *A*; G. B : group *B*; G. C : group *C*; and G. D : group *D*. (d) A special phenomenon was noticed; after the third injection (day 24), the rabbit ear of group *A* and group *B* was slouched (left) and the rabbit ear of group *C* and *D* became erected again (right). (e) On day 27, after the injection procedure, the HSs were harvested for further experiments. The numbers 0 to 3 represent group *A* to *D*, respectively.

**Figure 2:** Morphology analysis of hypertrophic scars after *Galangin* injection. (a) HE staining showed different protuberant degrees among these groups. (b) The SEI was measured according to the observation of HE staining. The SEI significantly decreased in group *C* and *D*. ^*∗*^*P* < 0.05, compared with the control group (saline injection). (c) Masson staining revealed the collagen and arrangement in the HS tissues.

**Figure 3:** Representative immunohistochemical staining of (a) type I and (b) type III collagens, (c) TGF-*β*1, and (d) Smad 7 in each group.

**Figure 4:** The protein expression levels of type I and type III collagens, TGF-*β*1, and Smad 7. The protein levels were analyzed by western blot, and *β*-actin was used as an internal control. The representative and quantitative results of (a) type I and (b) type III collagens, (c) TGF-*β*1, and (d) Smad7 are shown. ^*∗*^*P* < 0.05, compared to the control group.

**Figure 5:** The effect of *Galangin* on the mRNA expression of (a) type I collagen, (b) type III collagen, (c) TGF-*β*1, and (d) Smad 7. The mRNA expression was detected with real-time PCR and normalized to that of GADPH. The horizontal bar indicates the mean of the measurements in each group. ^*∗*^*P* < 0.05, compared to the control group.

**Table 1:** Primer sequences for PCR amplification.

Gene		Sequence (5′-3′)
Collagen I	Forward:	AAG GAG ACA CTG GTG CCA AG
	Reverse:	AGT AGG TCC GGG TTC ACC TC

Collagen III	Forward:	TGG GAA GCC AGG AGT TAA TG
	Reverse:	ATC CAG GGT TTC CGT CTC TT

TGF-*β*1	Forward:	CCA GGA ATA CAG CAA CGA TTC C
	Reverse:	CCA CTG CCT CAC AAC TCC A

Smad 7	Forward:	GTG GCA TAC TGG GAG GAG AA
	Reverse:	TTG TTG TCC GAA TTG AGC TG

GAPDH	Forward:	ATT TGA AGG GCG GAG CCA AA
	Reverse:	TCA TGA GCC CCT CCA CAA TG

## Data Availability

The data used to support the findings of this study are available from the corresponding author upon request.
